The article "Influence of Diagnostic Informing on Negative Emotions, Illness Perception, Self-Perceived Burden, and Posttraumatic Stress Disorder in Patients with Gastrointestinal Tumors" was retracted in 2023. Reasons: unreliable results or conclusions; lack of ethics approval or compliance; concerns about the data; concerns about the peer review.

# Influence of Diagnostic Informing on Negative Emotions, Illness Perception, Self-Perceived Burden, and Posttraumatic Stress Disorder in Patients with Gastrointestinal Tumors

**DOI:** 10.1155/2021/2568195

**Published:** 2021-10-13

**Authors:** Wei Xu, Juan Tang, Jie Chen

**Affiliations:** ^1^Nursing Department, Pingxiang Hospital of Southern Medical University, Pingxiang, Jiangxi 337000, China; ^2^Department of Oncology, Pingxiang Hospital of Southern Medical University, Pingxiang, Jiangxi 337000, China; ^3^Department of Science and Education, Pingxiang Hospital of Southern Medical University, Pingxiang, Jiangxi 337000, China

## Abstract

**Objective:**

To investigate the influence of diagnostic informing on negative emotions, illness perception (IP), self-perceived burden (SPB), and posttraumatic stress disorder (PTSD) in patients with gastrointestinal tumors.

**Methods:**

A total of 261 patients with gastrointestinal tumors admitted to our hospital from January 2018 to December 2020 were selected. According to whether the patients were informed of the disease diagnosis, they were divided into the informing group (*n* = 125) and the concealment group (*n* = 136). The self-rating anxiety scale (SAS), the self-rating depression scale (SDS), the brief illness perception questionnaire (BIPQ), the self-perceived burden scale (SPBS), and the PTSD checklist-civilian version (PCL-C) were used to investigate the two groups.

**Results:**

The SAS and SDS scores of the informing group were lower than those of the concealment group (*t* = 7.853 and 6.444, *P* < 0.05). The total BIPQ score of the informing group was higher than that of the concealment group (*t* = −4.089, *P* < 0.05). The total SPBS score of the informing group was lower than that in the concealment group (*t* = 2.443, *P* < 0.05). The total PCL-C score of the informing group was lower than that of the concealment group (*t* = 2.173, *P* < 0.05).

**Conclusion:**

Diagnosis informing can reduce the negative emotions, increase positive IP, and reduce the risk of SPB and PTSD in patients with gastrointestinal tumors.

## 1. Introduction

Gastrointestinal tumor is a tumor occurring in the stomach and intestine, mainly including gastrointestinal adenoma, fibroma, gastric cancer, and colorectal cancer. It has the characteristics of rapid progress and high mortality rate and has become a frequent clinical disease [1]. There is no obvious manifestation in the initial stage of the disease, but with the progress of the disease, symptoms such as abdominal pain, hematemesis, melena, and intestinal obstruction may appear and even lead to multiple organ failure, which is life-threatening and has a great impact on the quality of life of patients [2]. At present, surgery, chemotherapy, radiotherapy, and traditional Chinese medicine therapy are common clinical tumor treatments, which have a certain effect on patients with gastrointestinal tumors and can improve the prognosis of patients [3]. In recent years, with the continuous improvement of the social level, the survival time of tumor patients has been prolonged, and the psychological status of patients has gradually become the focus of clinical observation.

The article "Influence of Diagnostic Informing on Negative Emotions, Illness Perception, Self-Perceived Burden, and Posttraumatic Stress Disorder in Patients with Gastrointestinal Tumors" was retracted in 2023. Reasons: unreliable results or conclusions; lack of ethics approval or compliance; concerns about the data; concerns about the peer review.

Diagnosis informing is a strong psychological shock, which can cause a variety of emotional disorders and psychological problems, resulting in endocrine disorders and metabolic and immune dysfunction and affecting the disease progression, treatment, recovery, and outcome of patients [4]. Anxiety is a form of psychological stress protection mechanism generated by patients' excessive worry in the case of emergency or expected adverse outcomes, which can cause irritability, panic, and other emotions and result in inattention and memory reduction [5]. Depression is a kind of bad psychology characterized by low spirit, slow thinking, and decreased willpower activity. It can gradually progress from low emotion to grief-stricken, negative pessimistic, and extreme thoughts such as suicide which may occur in severe cases [6]. Illness perception (IP) is a process in which patients explain the current symptoms through the disease knowledge and experience they have acquired, thus forming stress responses to their own disease cognition and understanding [7]. Self-perceived burden (SPB) refers to patients' feelings of guilt, pain, concern, worry, and other feelings that are caused by their own diseases and the negative impact of care needs on the caregivers [8]. Posttraumatic stress disorder (PTSD) is a delayed stress response in patients after severe trauma. It is caused by the stressors of death-threatening events, severe violence, psychological trauma, and other traumatic events, and the clinical symptoms are progressive and lifelong [9].

According to medical ethics, medical staff informing patients of the diagnosis truth is an act of respecting patients' right to life and right to know. However, the traditional culture of China does not advocate informing patients about the diagnosis information of the disease. In order to avoid the severe blow of the patients, most family members of patients are not willing to let the patients know the true condition of the disease and often require medical staff to conceal the diagnosis of the patients or only inform the patients of part of the disease [10]. McPherson et al. [11] conducted an investigation on 57 stroke patients and found that the proportion of doctors informing patients of the true situation was as high as 90.0%. Jie et al. [12] reported that about 60.5%–98.0% of patients with liver cancer thought they should know the diagnosis. Goldfarb et al. [13] believed that, for patients with Alzheimer's disease and related dementia, even if the patient has great difficulty in receiving a diagnosis, timely disclosure of the diagnosis and the implementation of psychological education to patients is beneficial for patients and medical staff. Diagnosis informing is beneficial to increase the possibility of patients participating in decision-making and planning for the future, reduce potential risk factors of the disease, and reduce clinical symptoms. Dunham's team [14] observed and studied 8 patients with dementia and found that informing the diagnosis is an overwhelming and highly stressful event for patients with dementia, which may cause patients to have a higher stress response, and that the notification of the diagnosis of dementia may be associated with the symptoms of PTSD. At present, whether it is necessary to inform patients of the truth of diagnosis is a difficult problem faced by medical staff and their families, and there is not enough clinical research evidence. Therefore, this study aimed to investigate the effects of diagnostic notification on negative emotions, IP, SPB, and PTSD in patients with gastrointestinal tumors.

The article "Influence of Diagnostic Informing on Negative Emotions, Illness Perception, Self-Perceived Burden, and Posttraumatic Stress Disorder in Patients with Gastrointestinal Tumors" was retracted in 2023. Reasons: unreliable results or conclusions; lack of ethics approval or compliance; concerns about the data; concerns about the peer review.

## 2. Subjects and Methods

### 2.1. Subjects

A total of 261 patients with gastrointestinal tumors admitted to Pingxiang People's Hospital from January 2018 to December 2020 were selected. The inclusion criteria were as follows: age ≥ 18 years; basic understanding of expression skills; available for review on time. The exclusion criteria were as follows: people with other serious systemic diseases; people with mental illness; people who died during the study; people who withdrew midway. The patients were divided into the informing group (*n* = 125) and the concealment group (*n* = 136) according to whether they were informed of the disease diagnosis. In the informing group, the diagnosis of gastrointestinal tumor was informed by the doctor or family member. There were 70 males and 55 females, and they were aged from 26 to 72 years, with an average age of 49.16 ± 10.38 years; education level: 31 cases of primary school or below, 55 cases of junior middle school, and 39 cases of senior high school or above. In the concealment group, the doctors and family members informed the diagnosis of gastrointestinal benign diseases (appendicitis, intestinal obstruction, gastric ulcer perforation, gastrointestinal hemorrhage, etc.) and concealed the diagnosis of gastrointestinal tumor. There were 73 males and 63 females, and they were aged from 25 to 74 years, with an average age of 50.21 ± 9.75 years; education level: 34 cases of primary school or below, 60 cases of junior middle school, and 42 cases of senior high school or above. There was no significant difference in general data between the two groups (*P* > 0.05), indicating comparability. This study was approved by the Ethics Committee, and the informed consent form was signed by the patient or his/her family.

The article "Influence of Diagnostic Informing on Negative Emotions, Illness Perception, Self-Perceived Burden, and Posttraumatic Stress Disorder in Patients with Gastrointestinal Tumors" was retracted in 2023. Reasons: unreliable results or conclusions; lack of ethics approval or compliance; concerns about the data; concerns about the peer review.

### 2.2. Methods

When the diagnosis was notified, family members should choose a quiet and comfortable environment with a certain degree of privacy. The data were obtained by a combination of questionnaire and semistructured interview. On the day of discharge, the patient's family members and the doctor in charge were asked to confirm whether the patient had been informed of the disease diagnosis. The specific situation in the process of diagnosis notification mainly included the following: whether to inform, whom to inform, time to inform, place to inform, content to inform, extent to inform, and family members' suggestions to inform. The research scale was used to investigate the patients. During the study, the researchers did not implement any intervention measures, but only carried out the investigation and study. Questionnaires were filled out under the guidance of uniformly trained researchers, indicating the purpose and matters need attention of the study. A total of 261 questionnaires were sent out, and 261 were effectively taken back. After the questionnaires were returned, they were checked by two people. After the questionnaire was filled in, the patient's family members were invited to interview, and the researcher himself recorded the key points on the spot. After the interview, the interviewer immediately supplemented and sorted out the interview records.

### 2.3. Tool

#### 2.3.1. Self-Rating Anxiety Scale (SAS) and Self-Rating Depression Scale (SDS) [15, 16]

There were 20 items in the SAS, using a 4-level scoring system, with 15 positive scores and 5 negative scores. No anxiety: <50 points, mild anxiety: 50–59 points, moderate anxiety: 60–69 points, and severe anxiety: ≥70 points. The higher the score, the more severe the anxiety. Cronbach's *α* coefficient of the scale was 0.824.

There were 20 items in the SDS, using a 4-level scoring system, with 10 positive scores and 10 negative scores. No depression: <53 points, mild depression: 53–62 points, moderate depression: 63–72 points, and severe depression: ≥73 points. The higher the score, the more severe the depression. Cronbach's *α* coefficient of the scale was 0.895.

The article "Influence of Diagnostic Informing on Negative Emotions, Illness Perception, Self-Perceived Burden, and Posttraumatic Stress Disorder in Patients with Gastrointestinal Tumors" was retracted in 2023. Reasons: unreliable results or conclusions; lack of ethics approval or compliance; concerns about the data; concerns about the peer review.

#### 2.3.2. Brief Illness Perception Questionnaire (BIPQ) [17]

There were 9 items in the BIPQ, and the first 8 items were scored by 0–10 points, which included the impact of the disease on life, the time the patient thinks the disease will last, the self-control over the disease, the patient's perception of the treatment effect, the size of the symptoms caused by the disease, the degree of care for the disease, the knowledge of the disease, and the degree of emotional impact. The higher the score, the better the illness perception. Item 9 was an open question about etiological cognition. Cronbach's *α* coefficient of the scale was 0.770.

#### 2.3.3. Self-Perceived Burden Scale (SPBS) [18]

There were 21 items in the SPBS, including financial/family burden, mood/emotional burden, care burden, and treatment burden. A 5-level scoring system was used. No SPB: <30 points, mild SPB: 30–50 points, moderate SPB: 50–70 points, and severe SPB: ≥70 points. The higher the score, the heavier the SPB. Cronbach's *α* coefficient of the scale was 0.938.

#### 2.3.4. PTSD Checklist-Civilian Version (PCL-C) [19]

There were 17 items in PCL-C, which were divided into reexperience, avoidance/numbness, and hypervigilance. The 5-level scoring method was adopted. The total score > 38 points was positive for PTSD. The higher the score, the more severe the PTSD symptoms. Cronbach's *α* coefficient of the scale was 0.822. Traumatic events were defined as hospitalization and treatment due to gastrointestinal disease.

### 2.4. Statistical Analysis

Data were processed by SPSS 22.0. The quantitative data were expressed as “mean ± standard deviation” ($\bar{x}\pm s$), and the *t*-test was used for comparison. Differences were considered statistically significant at *P* < 0.05.

## 3. Results

### 3.1. Comparison of Negative Emotions between Two Groups

The SAS and SDS scores of the informing group were lower than those of the concealment group, with statistical significance (*t* = 7.853 and 6.444, *P* < 0.05), as shown in Table 1.

### 3.2. Comparison of IP between Two Groups

The total BIPQ score of the informing group was higher than that of the concealment group, with statistical significance (*t* = −4.089, *P* < 0.05), as shown in Table 2.

### 3.3. Comparison of SPBS between Two Groups

The total SPBS score of the informing group was lower than that in the concealment group, with statistical significance (*t* = 2.443, *P* < 0.05), as shown in Table 3.

### 3.4. Comparison of PTSD between Two Groups

The total PCL-C score of the informing group was lower than that of the concealment group, with statistical significance (*t* = 2.173, *P* < 0.05), as shown in Table 4.

The article "Influence of Diagnostic Informing on Negative Emotions, Illness Perception, Self-Perceived Burden, and Posttraumatic Stress Disorder in Patients with Gastrointestinal Tumors" was retracted in 2023. Reasons: unreliable results or conclusions; lack of ethics approval or compliance; concerns about the data; concerns about the peer review.

## 4. Discussion

Gastrointestinal tumors, as a serious disease, can cause digestive function decline and immune function decline of patients and endanger the life safety of patients. Effective treatment is of great significance for patients with gastrointestinal tumors, which can alleviate the gastrointestinal symptoms and increase the chance of recovery [20]. Tumor is a kind of malignant psychological stimulation closely related to the emotional changes of patients. Once the patients know about it, they may produce a variety of adverse emotions and increase psychological trauma, but at the same time, it may enable the patients to master their own situation and improve coordination. Jie et al. [21] reported that 88.1% of patients with liver cancer had the intention to know the actual situation, but only 52.6% of patients were informed of the actual situation. At present, there is no unified consensus on whether to inform patients of the diagnosis.

Anxiety and depression are the main components of negative emotions, and IP is the stress response of patients to perceive the threat of their own diseases, both of which are correlated with the occurrence and development of diseases. Niemier [22] believed that it is often difficult to inform the elderly about the diagnosis of cancer, but regardless of the clinical situation, patients should be informed of the diagnosis of tumor disease step by step through reasonable methods. Mormont's team [23] conducted a survey of 44 Alzheimer's disease patients and found that being told that the disease rarely or never causes harm to the patient, the patient often does not become hostile to the medical staff, and the diagnosis notification can alleviate the bad mood of the patient. In this study, the SAS and SDS scores of the informing group were lower than those of the concealment group. The total score of the BIPQ in the informing group was higher than that in the concealment group, and the patients had a higher degree of personal control, symptom identification, disease understanding, and lower emotional response. The results showed that diagnosis informing can reduce the negative emotions of patients with gastrointestinal tumors and increase the positive IP. We think the reason for this conclusion is that medical staff proactively inform patients of the diagnosis and can appropriately provide patients with effective information, and they can take the initiative in clinical decision-making and control the patients' health, participate in the process of clinical treatment and reexamination, actively cooperate with the medical staff to take corresponding measures, freely vent their emotions, and obtain the comfort of their families, thereby reducing negative emotions and promoting the improvement of the disease. In addition, after patients know the diagnosis, they can communicate with physicians on the treatment of the disease, timely solve the existing confusion and problems, and increase the patients' sense of control over personal conditions. Moreover, patients have a clear goal to obtain disease-related information, which is conducive to identifying clinical symptoms and understanding the occurrence and development of the disease. At the same time, the diagnosis informing can alleviate the adverse emotions of patients, establish confidence in treatment, and enable patients to form an optimistic attitude [24].

The article "Influence of Diagnostic Informing on Negative Emotions, Illness Perception, Self-Perceived Burden, and Posttraumatic Stress Disorder in Patients with Gastrointestinal Tumors" was retracted in 2023. Reasons: unreliable results or conclusions; lack of ethics approval or compliance; concerns about the data; concerns about the peer review.

This study showed that the total SPBS score of the informing group was lower than that of the concealment group. This suggested that diagnosis informing may reduce SPB in patients with gastrointestinal tumors. Affected by factors such as economy, mood, care, treatment, and other factors, patients with tumor often worry that their diseases are a burden for others and find it difficult to accept the occurrence of diseases, resulting in guilt, pain, and other feelings. Giving reasonable diagnosis information to patients can strengthen communication between patients and their families and physicians, control disease progression, reduce psychological pressure, and eliminate the sense of burden. In addition, the study found that the total PCL-C score in the informing group was lower than that in the concealment group. The results suggested that diagnosis informing can reduce the risk of PTSD in patients with gastrointestinal tumors. As a traumatic event, patients with tumor have severe mental stress. After experiencing the disease, they usually have strong negative psychology, are worried about the disease progression or deterioration again, and are afraid of the impact on life safety, thus causing PTSD. Patients with gastrointestinal tumor who know the truth of the diagnosis often have accepted their own diseases after they are discharged from the hospital, but concealing the diagnosis may interfere with the natural recovery of PTSD, causing patients to have PTSD for a long time or even lifelong stress symptoms [25].

In addition, doctors or family members using the correct method to inform the diagnosis can make the patient better accept the disease and more actively cooperate with treatment. In the process of notification, medical staff should gradually disclose the diagnosis of the disease from the shallower to the deeper and selectively inform the patient according to the specific situation of the patient or according to the requirements of the family members. After being informed of the diagnosis, the doctor can explain the details of the treatment process to the patient and their family members in an easy-to-understand language and provide psychological counseling to the patient so that the patient can actively face the disease and establish an optimistic attitude.

The article "Influence of Diagnostic Informing on Negative Emotions, Illness Perception, Self-Perceived Burden, and Posttraumatic Stress Disorder in Patients with Gastrointestinal Tumors" was retracted in 2023. Reasons: unreliable results or conclusions; lack of ethics approval or compliance; concerns about the data; concerns about the peer review.

## 5. Conclusion

In summary, diagnosis informing can reduce the negative emotions, increase positive IP, and reduce the risk of SPB and PTSD in patients with gastrointestinal tumors. Therefore, medical staff should cooperate together with family members to inform patients of diagnosis results at an appropriate time and in an appropriate way according to the individual conditions of patients, so as to promote their physical and mental health. The shortcomings of this study are the small sample size and the limitations of cultural background. The results need to be further confirmed by expanding the sample size and considering cultural differences in the future.

## Figures and Tables

**Table 1:** Comparison of negative emotions between two groups (*n*, $\bar{x}$ ± *s*, scores).

Items	The informing group (*n* = 125)	The concealment group (*n* = 136)	*t* value	*P* value
SAS	49.83 ± 4.76	54.70 ± 5.22	7.853	≤0.001
SDS	51.58 ± 5.03	56.19 ± 6.38	6.444	≤0.001

**Table 2:** Comparison of IP between two groups (*n*, $\bar{x}$ ± *s*, scores).

Items	The informing group (*n* = 125)	The concealment group (*n* = 136)	*t* value	*P* value
Disease influence	6.79 ± 2.34	6.85 ± 2.16	0.215	0.829
Disease process	6.54 ± 2.20	6.68 ± 2.27	0.505	0.614
Personal control	7.91 ± 2.06	5.13 ± 1.92	−11.284	≤0.001
Treatment control	6.23 ± 2.15	6.46 ± 2.18	0.857	0.392
Symptom recognition	7.37 ± 1.69	5.37 ± 2.04	−8.583	≤0.001
Disease attention	8.02 ± 1.58	7.88 ± 1.35	−0.771	0.441
Disease awareness	8.11 ± 1.30	6.26 ± 1.93	−9.002	≤0.001
Emotional response	4.28 ± 2.46	5.01 ± 2.57	2.339	0.020
Total BIPQ score	55.25 ± 10.73	49.64 ± 11.38	−4.089	≤0.001

**Table 3:** Comparison of SPBS between two groups (*n*, $\bar{x}$ ± *s*, scores).

Items	The informing group (*n* = 125)	The concealment group (*n* = 136)	*t* value	*P* value
Financial/family burden	16.28 ± 5.91	18.46 ± 5.74	3.022	0.003
Mood/emotional burden	14.03 ± 4.11	14.72 ± 3.85	1.400	0.162
Care burden	10.52 ± 4.56	11.13 ± 4.39	1.101	0.272
Treatment burden	8.74 ± 3.46	9.60 ± 3.55	1.978	0.049
Total SPBS score	49.57 ± 16.02	53.91 ± 12.59	2.443	0.015

**Table 4:** Comparison of PTSD between two groups (*n*, $\bar{x}$ ± *s*, scores).

Items	The informing group (*n* = 125)	The concealment group (*n* = 136)	*t* value	*P* value
Reexperience	9.58 ± 4.47	10.15 ± 4.38	1.040	0.299
Avoidance/numbness	11.61 ± 5.23	12.77 ± 6.01	1.657	0.098
Hypervigilance	10.24 ± 4.18	11.45 ± 5.29	2.038	0.043
Total PCL-C score	31.43 ± 11.05	34.37 ± 10.80	2.173	0.031

The article "Influence of Diagnostic Informing on Negative Emotions, Illness Perception, Self-Perceived Burden, and Posttraumatic Stress Disorder in Patients with Gastrointestinal Tumors" was retracted in 2023. Reasons: unreliable results or conclusions; lack of ethics approval or compliance; concerns about the data; concerns about the peer review.

## Data Availability

The data used and/or analyzed during the current study are available from the corresponding author upon request.
